# Adjuvant Application of Shenmai Injection for Sepsis: A Systematic Review and Meta-Analysis

**DOI:** 10.1155/2022/3710672

**Published:** 2022-08-09

**Authors:** Ye Sun, Yilin Liu, Li Li, Bing Xue, Yan Cao

**Affiliations:** ^1^Department of Critical Care Medicine, Yuebei People's Hospital, Shaoguan 512000, Guangdong, China; ^2^General Practice Department, Yuebei People's Hospital, Shaoguan 512000, Guangdong, China

## Abstract

**Objective:**

To compare the efficacy and safety of Shenmai injection plus regular treatment versus regular treatment alone in the treatment of sepsis.

**Methods:**

Review Manager 5.3 was used. Databases including PubMed, Cochrane Library, Wan-FANG, VIP, CNKI, and CBM were searched for the relative control and randomized studies till June 2022. Primary outcomes were 28-day mortality; case fatality rate; APACHE II score; and levels of procalcitonin, tumor necrosis factor-*α*, interleukin-6, and C-reaction protein. Secondary outcomes were measurements related to inflammatory reactions, coagulation function, immune function, and organ function.

**Results:**

In total 21 studies with 1469 patients were included. Shenmai injection plus regular treatment of sepsis significantly decreased 28-day mortality rate (odds ratio: 0.36 (0.20, 0.63); *p*=0.0004) and case fatality rate (odds ratio: 0.32 (0.19, 0.54), *p* < 0.0001) and significantly further reduced APACHE II score (standard mean deviation: −1.14 (−1.30, 0.99); *p* < 0.00001). Procalcitonin reduction was similar in the two groups (standard mean deviation: −0.59 (−1.64, 0.46); *p*=0.27). Tumor necrosis factor-*α* (standard mean deviation: −1.96 (−2.79, −1.13); *p* < 0.00001), interleukin-6 (standard mean deviation: −1.52 (−2.13, −0.91); *p* < 0.00001), and C-reaction protein (standard mean deviation: −2.37 (−4.26, −0.49); *p*=0.01) levels were significantly further decreased in the Shenmai injection group. Most of the measurements related to inflammatory reaction, coagulation function, immune function, and organ function were significantly regulated in the Shenmai injection group. Furthermore, there was no adverse event, and two study groups had similar adverse event rates.

**Conclusion:**

Shenmai injection as adjuvant therapy shall be effective and safe in the treatment of sepsis. However, further investigation is still warranted especially regarding safety. Adjuvant application of Shenmai injection in sepsis is worth further investigation.

## 1. Introduction

Sepsis refers to life-threatening organ dysfunction induced by the host response to infection disorders [1]. It is one serious complication among intensive care unit (ICU) patients affected by infection, shock, burn, etc. Sepsis accounted for 10%–40% of ICU cases [2], and the global incidence of sepsis is increasing 2%–9.5% each year [3]. This trend was mainly attributed to old age, immune suppression, and multiple resistant bacteria [3]. Morality rates of sepsis patients ranged from 20% to 50% [3–6]. In Western countries, it is a leading cause of ICU death only secondary to coronary heart disease [2]. Current treatment options for sepsis include early fluid resuscitation, anti-infection, vasoactive agent usage, protective ventilation strategy, hemopurification, etc. However, the poor prognosis of sepsis patients makes sepsis treatment still a challenge. It is necessary to develop a novel treatment strategy or option. Traditional Chinese medicine (TCM) has accumulated certain understanding and treatment experience for sepsis. Therefore, TCM treatment methods are receiving more and more attention from domestic and international researchers.

Shenmai injection was a Chinese patent drug widely used as adjuvant therapy for sepsis in Chinese hospitals in recent decades. It was prepared with ginseng and Ophiopogon. The formula of Shenmai injection was modified from Sheng Mai San recorded in Qian Jing Yao Fang of the Tang Dynasty [7]. In TCM, this formula has the effect of enhancing qi, nourishing fluid, replenishing vital energy, promoting blood circulation, dispersing phlegm, etc. The major components of Shenmai injection include ginsenoside saponins, ophiopogon saponin, ophiopogon flavonoids, ginseng polysaccharides, and ophiopogon polysaccharides. Previous studies demonstrated that ginsenoside had an immune regulation activity that could improve the suppression of cyto-immune function in burn sepsis [8]. Ginsenoside has the obvious anti-inflammation effect that it could downregulate the levels of tumor necrosis factor (TNF-*α*), interleukin-1 (IL-1), IL-6, IL-8, IL-10, and nitric oxide (NO) [9]. It was also revealed that Shenmai injection could inhibit over-releasing of inflammatory mediators, reduce inflammatory reaction, clear free radical, regulate immune function, enhance cyto-metabolism, prevent shock and cardiac arrhythmia, have cardiotonic action, improve hemorheology, and prevent aging [10].

There has been a number of studies investigating Shenmai injection in the treatment of sepsis, most of which were published in Chinese journals. However, there is no related meta-analysis to provide pooled evidence regarding this issue. Therefore, we performed the present meta-analysis in order to evaluate the efficacy and safety of Shenmai injection as adjuvant therapy in the treatment of sepsis, which might provide an access for the domestic and international researchers to know about the application of Shenmai injection in sepsis.

## 2. Method and Materials

### 2.1. Inclusion and Exclusion Criteria

The inclusion criteria were as follows: (1) types of studies: randomized controlled studies; (2) types of participants: patients with sepsis following the diagnosis criteria of sepsis defined by the International Sepsis Definition Conference of 2001 [11]; (3) intervention: the patients in the control group only received regular Western treatment for sepsis, and the patients in the experimental group received regular Western treatment combined with Shenmai injection; regular treatment of sepsis may include fluid resuscitation, anti-infection, serum sugar control, maintenance of homeostatic equilibrium, mechanical ventilation, and comprehensive therapy such as nutrition support and administration of glucocorticoids. Treatment length is at least 7 days; (4) outcome and measurements: primary outcome included APACHE II score, 28-day mortality rate, case fatality rate, procalcitonin (PCT) levels, TNF-*α* levels, IL-6 levels, and C-reaction protein (CRP) levels. The included study had at least one primary outcome.

Exclusion criteria were as follows: (1) retrospective or observational studies and animal studies were excluded; (2) for the experimental group, only Shenmai injection was added to the regular Western treatment, regardless of administration methods. No other treatment such as electroacupuncture, acupoint application, or other Western drugs or TCM was used; (3) if the results of one study were divided into multiple articles, only one article with the relatively complete result was included and the rest articles were excluded.

### 2.2. Article Retrieval

The studies investigating Shenmai injection as adjuvant therapy in the treatment of sepsis till June 2022 were retrieved using English and Chinese databases. The English databases included PubMed and Cochrane Library. The Chinese databases included Wan-Fang, VIP, CNKI, and CBM. The retrieval terms were “sepsis”, “Shenmai injection”. The Chinese retrieval terms were corresponding to Chinese for the retrieval terms above. The references of important articles were also manually retrieved.

### 2.3. Literature Screening, Data Extraction, and Quality Assessment

Literature screening and data extraction were performed by two independent reviewers respectively. During literature screening, duplication, title, abstract, and main text were examined. The situation that data of one study were separately published in multiple articles was also examined. Only the article containing the most complete data was included for further examination. The results of literature screening and data extraction by the two reviewers were compared, discussed, and determined. When necessary, a third experienced reviewer was invited. The extracted data included author name, publishing year, sample size, patient age, intervention in experimental group and control group, treatment length, and multiple outcome measurements.

Cochrane risk of bias tool was used for quality assessment of the included studies. The assessment items were random sequence generation, allocation concealment, blinding of participants and personnel, blinding of outcome assessment, incomplete outcome data, and selective reporting. Each item was rated as low, unclear, and high risk.

### 2.4. Outcome Measurements

The primary outcome measurements included 28-day mortality rate; case fatality rate; APACHE II score; and levels of PCT, CRP, IL-6, and TNF-*α*. The secondary outcome measurements included the following: immune function: CD3, CD4, CD8, CD4/CD8, and natural killer (NK); organ function: alanine transaminase (ALT), aspartate transaminase (AST), blood urea nitrogen (BUN), creatinine (Cr), lactate dehydrogenase (LDH), creatine kinase (CK), creatine kinase isoenzyme-MB (CK-MB), B-brain natriuretic peptide (BNP), and troponin I (TnI); coagulation function: activated partial thromboplastin time (APTT), prothrombin time (PT), thrombin time (TT), fibrinogen (FIB), platelet (PLT), and D-Dimer (D-D); inflammation factors: IL-6, IL-1*β*, and IL-8; other measurements: white blood cell (WBC) and hemoglobin (Hb). Except 28-day mortality rate and case fatality rate, the alteration from the baseline of the rest variables was compared between the two groups. For example, APACHE II score alteration = APACHE II score after treatment − APACHE II score at baseline. A positive value indicated APACHE II score increased, whereas a negative value indicated APACHE II score decreased.

### 2.5. Statistical Analysis

The statistical analysis was performed using the statistical software Review Manager 5.3. Odds ratios (ORs) for categorical variables were calculated; weighted mean difference (WMD) for numerical data was calculated; all effect sizes were expressed with a 95% confidence interval (95% CI). If different units were used for continuous variables in included studies, standard mean difference (SMD) was used for comparison. The heterogeneity test was performed using a standard chi-squared (*I*^2^*Q*) test. If *p* > 0.1, *I*^2^ < 50%, the fixed effect model was used; if *p* > 0.1, *I*^2^ > 50%, the random effect model was used. When heterogeneity was significant, a sensitivity test was performed. In the sensitivity test, studies were ruled out one by one. If the heterogeneity result was not changed, the result was stable. If the result was changed, the study identified could greatly impact the result and it was closely studied to further determine the source of heterogeneity. For the analysis including no less than 10 studies, a funnel plot was used to estimate the publication bias.

## 3. Results

### 3.1. Literature Screening Result and Characteristics of the Included Studies

In total, 38 articles were retrieved from the databases mentioned above, 30 studies were retrieved from CNKI, 26 from CBM, 28 from VIP, 22 from Wan-Fang, and 0 from PubMed and Cochrane library. After examination of duplication and situation of multiple articles from one study, 8 articles were excluded. After examination of the title and abstract, 5 articles were excluded. After the main text examination, 4 articles were excluded, and 21 studies were finally included in the present meta-analysis. The study selection process is shown as a flowchart in Figure 1.

The characteristics of included studies are summarized in Table 1 [12–32]. In total, 21 studies with 1469 participants were included in this study. All studies were randomized controlled studies, and the baseline characteristics of patients were consistent without statistical difference between the experimental group and the control group. The time span was 2010–2021. The dosage of Shenmai injection ranged from 40 mg/d to 240 mg/d. The length of treatment ranged from 7 to 10 days.

### 3.2. Quality Assessment Result

Among the included studies, 6 studies reporting random number table methods [12, 14, 18, 20, 21, 26, 29] and 3 studies reporting simple random sampling methods [15, 16, 32] were rated as low risk regarding selection bias of sequence generation. The other studies only mentioned randomization and were rated as unclear risk. None of the studies reported follow-up as they only evaluated short-term efficacy. Five studies had provided description or data of adverse events [25–27, 29–31]. The blindness of allocation, participants, and assessment was not reported by all studies, so they were rated as unclear. All studies provided complete data regarding the variables mentioned in the study methods, so they were all rated as low risk. The quality assessment results are summarized in Figure 2 and Figure 3. The quality of included studies was not high.

### 3.3. Outcomes

#### 3.3.1. Rate of 28-Day Morality

In total, 6 studies were included in this study (Figure 4). The heterogeneity test indicated that the difference between included studies was not significant (*p*=0.81, *I*^2^ = 0%) and a fixed effect model was used. The analysis result indicated that the 28-day mortality rate of the Shenmai injection group was significantly lower than that of the control group (OR: 0.36 (0.20, 0.63); *p*=0.0004).

#### 3.3.2. Case Fatality Rate

In total, 8 studies with 586 participants were included in the present analysis (Figure 5). The heterogeneity test result indicated that there was no significant heterogeneity (*p*=0.97, *I*^2^ = 0%) and a fixed effect model was used. The analysis result indicated that the case fatality rate of the Shenmai injection group was significantly lower than that of the control group (OR: 0.32 (0.19, 0.54); *p* < 0.0001).

#### 3.3.3. APACHE II Score Reduction from Baseline

In total, 11 studies were included in the analysis of APACHE II score reduction, which included 810 participants. According to the heterogeneity test result (*p* < 0.00001, *I*^2^ = 79%), there was a significant difference between the included studies (Figure 6). A random effect model was used. The analysis result showed that the APACHE II score reduction of the Shenmai injection group was significantly higher than that of the control group (SMD: −1.14 (−1.30, −0.99); *p* < 0.00001). The sensitivity test was performed, and the significant heterogeneity was stable upon removing each study.

#### 3.3.4. PCT Level Reduction

In total, 5 studies including 428 participants were included in the present analysis (Figure 7). The heterogeneity test result indicated that there was a significant difference between the included studies (*p* < 0.00001, *I*^2^ = 96%). A random effect model was used. The PCT level of the Shenmai injection group was slightly further decreased compared with that of the control group but showed no significant difference (SMD: −0.59 (−1.64, 0.46); *p*=0.27). The sensitivity test indicated that the heterogeneity was stable.

#### 3.3.5. TNF-*α*

In total, 8 studies with 594 participants were included in the present analysis (Figure 8). The heterogeneity test result demonstrated that the difference between the included studies was significant (*p* < 0.00001, *I*^2^ = 94%). Random effect model was used. The analysis result indicated that the level of TNF-*α* in the Shenmai injection group was significantly further decreased compared with the control group (SMD: −1.96 (−2.79, −1.13); *p* < 0.00001). The sensitivity test demonstrated that the heterogeneity was stable.

#### 3.3.6. IL-6

In total, 7 studies including 544 participants were included in the present analysis (Figure 9). The heterogeneity test result indicated that the included studies were significantly different (*p* < 0.00001, *I*^2^ = 90%). Random effect model was used. The analysis result indicated that the IL-6 level in the Shenmai injection group was significantly further decreased compared with the control group (SMD: −1.52 (−2.13, −0.91); *p* < 0.00001). The sensitivity test suggested that the heterogeneity was stable.

#### 3.3.7. CRP

In total, 10 studies including 786 participants were included in the present analysis (Figure 10). The heterogeneity test indicated the included studies were significantly different (*p* < 0.00001, *I*^2^ = 99%). Random effect model was used. Analysis result indicated that CRP level in the Shenmai injection group was significantly further decreased compared with the control group (SMD: −2.37 (−4.26, −0.49); *p*=0.01). The sensitivity test suggested that the heterogeneity result was stable.

#### 3.3.8. Publication Bias

A funnel plot of the APACHE II score was adopted to estimate the publication bias (Figure 11). The asymmetry was not significant, indicating the publication bias is not obvious and its impact on analysis result can be ignored.

#### 3.3.9. Measurements Related to Immune Function, Coagulation Function, Inflammation Reaction, and Organ Function

Other measurements were also compared and the results are summarized in Table 2. The measurements associated with coagulation function included PT, TT, APTT, FIB, PLT, and D-D; the measurements associated with immune function included CD3, CD4, CD8, CD4/CD8, and NK; the measurements associated with inflammation factor included IL-1 and IL-8, besides TNF-*α* and IL-6 above; the measurements associated with organ function included ALT, AST, BUN, Cr, LDH, CK, CK-MB, BNP, and TnI; other measurements included WBC and Hb.

The analysis results indicated that the addition of Shenmai injection could significantly further decrease the levels of PT, TT, APTT, D-D, IL-8, LDH, CK, CK-MB, BNP, and TnI compared with regular treatment alone; the addition of Shenmai injection could significantly further increase the levels of FIB, PLT, CD3, CD4, and CD4/CD8; Shenmai injection addition could significantly reverse the elevation trend of ALT, AST, BUN, and Cr levels compared with regular treatment alone (all *p* < 0.05). Furthermore, the changes in CD8, NK, IL-1, and WBC levels were not significantly different between the two groups (all *p* > 0.05).

#### 3.3.10. Adverse Events

There were 5 studies that provided text description or clinical data of adverse events. Among them, 4 studies reported that there were no drug-related adverse events during the study [25–27, 29, 31]. The study performed by Yu Limei reported 2 cases of chest distress plus cardiopalm and 2 cases of hypoglycemia in the Shenmai injection group, and 3 cases of hypoglycemia in the control group [30].

## 4. Discussion

Shenmai injection is widely used as adjuvant therapy in the treatment of sepsis in China. There are a number of studies investigating Shenmai injection. Therefore, we performed the present meta-analysis to evaluate the efficacy and safety of Shenmai injection as adjuvant therapy in the treatment of sepsis.

Our analysis demonstrated that the addition of Shenmai injection to regular treatment of sepsis significantly decreased the 28-day mortality rate and case fatality rate and significantly further reduced the APACHE II score. Furthermore, there was no adverse event, and two study groups had similar adverse event rates. Therefore, Shenmai injection as adjuvant therapy shall be effective and safe in the treatment of sepsis.

In the early phase of sepsis, the immune system was over-activated, releasing of inflammatory mediators was out of control, and systemic inflammatory response syndrome was induced. TNF-*α*, IL-6, and CRP are the most important pro-inflammatory mediators or inflammatory markers in the process [33]. If the microorganism was not cleared efficiently, early inflammatory reaction in sepsis could activate coagulation system, initiate coagulation cascade reaction, inhibit fibrinolysis pathway, induce microcirculation disturbance, interfere blood and oxygen supply to tissues, and lead to organ dysfunction [34]. In summary, the pathogenesis of sepsis is an interaction result of immune reaction, inflammatory reaction, and coagulation reaction; organ dysfunction (MODS) and disseminated intravascular coagulation (DIC) are common complications developed in sepsis progression and are major causes of death by sepsis [35].

According to our study result, a combination of Shenmai injection further decreased PCT, TNF-*α*, IL-6, CRP, and IL-8 levels, which indicated Shenmai injection suppressed pro-inflammatory mediator releasing and decreased systematic inflammatory reactions. The levels of PT, TT, APTT, and D-D were further decreased and the levels of FIB and PLT were further increased in the Shenmai injection group, which indicated that Shenmai injection improved coagulation function. The levels of CD3, CD4, and CD4/CD8 were further increased in the Shenmai injection group, which indicated that Shenmai injection improved immune function. The levels of LDH, CK, CK-MB, BNP, and TnI were further decreased and the elevation trend of ALT, AST, BUN, and Cr was reversed in the Shenmai injection group, which indicated that Shenmai injection had multiple organ protection activity. The regulation activity of Shenmai injection on immune function [36], inflammation reaction [37–39], and hemorheology [40–42] and further protection on multiple organs [37, 42] by Shenmai injection had been elucidated by a large number of animal or clinical studies. Therefore, we may conclude that the beneficial impact of Shenmai injection on inflammatory reaction, immune function, coagulation function, and organ function might contribute to better treatment outcome in the Shenmai injection group.

The result of adverse events indicated Shenmai injection was safe, however, which was concluded based on quite incomplete safety data. Previous studies had monitored adverse events related to Shenmai injection. According to the study performed by Wen et al. among 1216 cases, the rate of adverse events by Shenmai injection was 0.82% [43]. The study performed by Wang et al. with 421 medical cases using Shenmai injection reported an adverse event rate of 3.6% [44]. The study by Wen et al. was performed in a TCM hospital where the usage of Shenmai injection would be more standardized. This might contribute to the lower adverse event rate. However, in our study, the adverse events were reported by only a small portion of included studies and the safety information was incomplete, so interpretation of safety of Shenmai injection should be cautious.

The current treatment outcome for sepsis is not very satisfying. Accompanying more and more understanding of complicated mechanism of sepsis, researchers are seeking for novel treatment options, such as immune regulation therapy. Shenmai injection has a nature origin so that it could solve the problem of overuse of antibiotics in sepsis treatment. It has multiple effects including immune regulation activity. The treatment guidance strategy of Shenmai in sepsis was targeting microorganisms, removing toxicity, and promoting vital energy at the same time, which is similar to the current investigation trend and could be a good complementary. Therefore, Shenmai injection is a good potential candidate for sepsis treatment and is worth further investigation. However, the complicated components and agent interaction of TCM shall be addressed, and suitable investigation methods need to be developed or applied.

This is the first meta-analysis evaluating the efficacy and safety of Shenmai injection as adjuvant therapy in sepsis treatment. This study not only evaluated the effect of Shenmai injection on major treatment outcomes, but also evaluated the effect of Shenmai injection on measurements related to coagulation function, immune function, and organ functions, thus it provided a relatively comprehensive assessment of effect of Shenmai on sepsis. However, there are still some limitations in this study. (1) Some well-established indicators for systematic assessment of efficacy in sepsis treatment were not included such as ICU stay/hospital stay, mechanical ventilation rates, and rate of multiple organ dysfunction syndrome (MODS), for most of the included studies did not report these measurements. (2) The quality of included studies was relatively poor: the randomization generation method was reported only by a small portion of the studies; blindness was not reported by all studies; and dropout was not well described. (3) Adverse events were not rigorously assessed. Adverse events are important in TCM assessment, but most of the included studies did not include adverse events into evaluation. Therefore, future relative clinical studies shall take these into consideration: inclusion of more well-established indicators; detailed information on study procedure; and a more complete and standard safety report.

Currently, the TCMs are mainly used within China and are known by very few physicians or researchers out of China. Moreover, some international medical journals' acceptance of the study of TCM is low due to the complicated components. Therefore, the researchers would intend to publish the studies on Shenmai injection in Chinese Medical Journals. Thus, the study quality and article writing followed a relatively lower standard. However, TCM is receiving more and more attention from international researchers, and this trend in the publication of TCM in Chinese Medical Journals is changing. When it comes to the credibility of the results, many studies are usually of lower quality, but they still can elucidate the efficacy and safety of Shenmai injection to a large extent. Moreover, Shenmai injection is widely used in Chinese hospitals, and there are several publications on Shenmai injection in sepsis in recent years which demonstrated that the efficacy and safety of Shenmai injection are recognized by Chinese physicians. Therefore, I think the relatively low quality of studies included in present analysis may lead to certain bias, but the analysis results and conclusion are still reliable.

## 5. Conclusion

Shenmai injection as adjuvant therapy shall be effective and safe in the treatment of sepsis. However, further investigation is still warranted, especially regarding the safety profile. Adjuvant application of Shenmai injection in sepsis is worth further investigation.

## Figures and Tables

**Figure 1:** Flowchart of the studies' selection process.

**Figure 2:** Risk of bias graph of included studies.

**Figure 3:** Summary of risk bias of included studies.

**Figure 4:** Forest plot of 28-day morality rate in sepsis patients receiving Shenmai injection plus regular treatment versus regular treatment alone.

**Figure 5:** Forest plot of case fatality rate in sepsis patients receiving Shenmai injection plus regular treatment versus regular treatment alone.

**Figure 6:** Forest plot of APACHE II score in sepsis patients receiving Shenmai injection plus regular treatment versus regular treatment alone.

**Figure 7:** Forest plot of PCT levels in sepsis patients receiving Shenmai injection plus regular treatment versus regular treatment alone.

**Figure 8:** Forest plot of TNF-*α* in sepsis patients receiving Shenmai injection plus regular treatment versus regular treatment alone.

**Figure 9:** Forest plot of IL-6 levels in sepsis patients receiving Shenmai injection plus regular treatment versus regular treatment alone.

**Figure 10:** Forest plot of CRP levels in sepsis patients receiving Shenmai injection plus regular treatment versus regular treatment alone.

**Figure 11:** Funnel plot of APACHE II score for the publication bias.

**Table 1:** Characteristics of included studies.

First author, year	Sample size (E/C)	Age	Intervention		Treatment course	Outcome
			Experimental	Control		
Bao Jifeng, 2015 [12]	112 (56/56)	60.34 ± 4.31 (23–85）	Patients with hypotension: regular treatment+SI 100 ml/d	Regular treatment	7 d	Coagulation: PT, TT, APTT, FIB, PLT, D-D
			Patients without hypotension: regular treatment+SI 60 ml/d			Immune: CD3, CD4, NK
						Inflammation：TNF-*α*, IL-1*β*, IL-6, IL-8, CRP
						Organ: ALT, AST, BUN, Cr, LDH, CK, CK-MB
Chen Tengfei, 2020 [13]	62 (28/34)	61–91/67–95	Regular treatment+SI 200 ml/d	Regular treatment	7 d	28-day mortality
						Inflammation: PCT, CRP
Chen Wei, 2017 [14]	80 (40/40)	69.15 ± 5.62/69.23 ± 5.44	Regular treatment+SI 40 ml/d	Regular treatment	10	28-day mortality, case fatality rate
Chen Yuzhi, 2015 [15]	50 (25/25)	71.84 ± 15.17/73.40 ± 9.5	Regular treatment+SI 100 ml/d	Regular treatment	5–7 d	Case fatality rate, APACHE II score
						Coagulation: APTT, PT, AT, D-D, FIB, PLT;
						WBC, HB
Feng Gang, 2019 [16]	66 (33/33)	62.14 ± 18.72/61.78 ± 17.33	Regular treatment+SI 24-hour continuous infusion 10 ml/h (240 ml/d)	Regular treatment	7 d	APACHE II score
						Inflammation: TNF-*α*, CRP, IL-6
He Cong, 2019 [17]	32 (16/16)	59.75 ± 8.66/61.19 ± 8.26	Regular treatment+SI 200 ml/d	Regular treatment	7 d	28-day mortality
						Organ: BNP, TnI, CK-MB
Huang Zengfeng, 2010 [18]	60 (30/30)	61.5 ± 8.7/60.8 ± 9.2	Regular treatment+SI 100 ml/d	Regular treatment	7 d	APACHE II
						Inflammation: TNF-*α*, IL-1*β*, IL-6, IL-8, IL-10
Liu Linlin 2012 [19]	63 (31/32)	60–89	Regular treatment+SI 40 ml/d	Regular treatment	7 d	28-day mortality rate
						Organ：CK-MB, BNP, Cr
						Coagulation: PA, APTT, Hb
Li Wansheng, 2018 [20]	100 (50/50)	58.93 ± 5.46/59.73 ± 5.13	Regular treatment+SI 60 ml/d	Regular treatment	7 d	APACHE II score
						Coagulation: PLT, FIB, APTT
Liu Wenyue, 2018 [21]	106 (53/53)	66.73 ± 4.8/67.04 ± 4.75	Regular treatment+SI 100 ml/d	Regular treatment	7 d	Case fatality rate; APACHE II score
						Organs: BNP, CK, CK-MB, TnI Immune: CD4+, CD8+, NK
Ning Xiaoping, 2011 [22]	60 (30/30)	56.9 ± 2.3 (23–78)	Regular treatment+SI 60 ml/d	Regular treatment	7 d	Case fatality rate, APACHE II score
						Organ: Cr
						Coagulation: PLT
Ning Xiaoping, 2012 [23]	60 (30/30)	58.2 ± 3.6	Patients with hypotension: regular treatment+SI 100 ml/d	Regular treatment	7 d	Inflammation: TNF-*α*, IL-1, CRP
			Patients without hypotension: regular treatment+SI 60 ml/d			
Shen Liming, 2014 [24]	46 (23/23)	67.2 ± 8.1/65.5 ± 7.9	Regular treatment+SI 100 ml/d	Regular treatment	7 d	Fatality rate, APACHE II score
						Inflammation: CD3, CD4, CD8, CD4/CD8, NK
Wang Baohua, 2021 [25]	84 (42/42)	55.87 ± 5.24/56.32 ± 4.58	Patients with hypotension: regular treatment +CBP+SI 60 ml/d	Regular treatment+CBP	7 d	APACHE II score, case fatality rate; AE
			Patients without hypotension: regular treatment +CBP+SI 100 ml/d			Inflammation: CRP, PCT
						Coagulation: PT, TT, APTT, D-D
Wang Sen, 2016 [26]	96 (48/48)	69.15 ± 5.24/68.94 ± 5.17	Patients without hypotension：regular treatment+SI injection 120 ml/d	Regular treatment	7 d	APACHE II score; AE
			Patients with hypotension：regular treatment+SI 200 ml/d			Inflammation: CRP, PCT, TNF-*α*
Xu Wei, 2017 [27]	60 (30/30)	68.56 ± 3.39/69.34 ± 2.57	Regular treatment+SI 50 ml/d	Regular treatment	7 d	AE
						Organ: BNP, CK-MB, TnI
Xu Xiaoyun, 2015 [28]	80 (40/40)	60.8 ± 9	Regular treatment+SI 24-hour continuous infusion 10 ml/h (240 ml/d)	Regular treatment	7 d	AE
						Organ: ALT, AST, BUN, Cr, CK, CK-MB
						Inflammation: CRP, PCT, TNF-*α*, IL-6, IL-8, WBC
Yao Yabin, 2017 [29]	82 (41/41)	54.12 ± 11.18/51.27 ± 11.35	Regular treatment+SI 100 ml/d	Regular treatment	7 d	Case fatality rate, APACHE II score; AE
Yu Limei, 2016 [30]	70 (35/35)	58.31 ± 3.21/59.12 ± 3.32	Regular treatment+SI 40 ml/d	Regular treatment	7 d	AE
						Inflammation: CRP, TNF-*α*, IL-1, IL-6
Zeng Dao, 2013 [31]	50 (25/25)	50 ± 2.5 (24–75)	Patients with hypotension: regular treatment+SI 100 ml/d	Regular treatment	10 d	AE
			Patients without hypotension: regular treatment+SI 60 ml/d			Inflammation: TNF-*α*, IL-6, CRP
Zhou Yuanshen, 2016 [32]	50 (25/25)	72.62 ± 12.53	Regular treatment+SI 100 ml/d	Regular treatment	7 d	28-day mortality rate; APACHE II score
						Coagulation：APTT, PT, D-D, FIB, PLT, WBC, Hb

*Note.* SI, Shenmai injection; AE, adverse events; CRP, C-reaction protein; IL-6, interleukin-6; NK, natural killer; ALT, alanine transaminase; AST, aspartate transaminase; BUN, blood urea nitrogen; Cr, creatinine; LDH, lactate dehydrogenase; CK, creatine kinase; CK-MB, creatine kinase isoenzyme-MB; APTT, activated partial thromboplastin time; PT, prothrombin time; TT, thrombin time; FIB, fibrinogen; PLT, platelet; D-D, D-dimer; IL-1, interleukin-1; TNF-*α*, tumor necrosis factor-*α*; IL-8, interleukin-8; WBC, white blood cell; Hb, hemoglobin; BNP, B-brain natriuretic peptide; TnI, troponin I. Regular treatment of sepsis may include fluid resuscitation, anti-infection, serum sugar control, maintenance of homeostatic equilibrium, mechanical ventilation, and comprehensive therapy such as nutrition support and administration of glucocorticoids.

**Table 2:** Summary of comparisons of relevant measurements among the sepsis patients receiving Shenmai injection plus regular treatment versus regular treatment alone.

Outcome	No. of studies	No. of participants	Heterogeneity		Statistical method	Effect estimates	
			*I* ^2^	*p*		Effect size (95% CI)	P value
*Coagulation function*							
PT	6	456	84%	<0.00001	SMD, Fixed	−1.35 (−1.55, −1.14)	<0.00001
TT	3	256	25%	0.27	SMD, Fixed	−1.76 (−2.05, −1.47)	<0.00001
APTT	6	419	88%	<0.00001	SMD, Random	−0.85 (−1.45, −0.25)	0.005
FIB	4	272	69%	0.02	SMD, Random	1.24 (0.76, 1.73)	<0.00001
PLT	6	432	90%	<0.00001	SMD, Random	1.05 (0.37, 1.73)	0.002
D-D	5	356	82%	0.0002	SMD, Random	−0.97 (−1.51, −0.43)	0.0005

*Immune function*							
CD3	2	158	0%	0.41	SMD, Fixed	0.58 (0.27, 0.90)	0.0003
CD4	2	152	0%	0.48	SMD, Fixed	0.97 (0.64, 1.31)	<0.00001
CD8	2	152	89%	0.003	SMD, Random	−0.51 (−1.57, 0.55)	0.35
CD4/CD8	2	158	25%	0.25	SMD, Fixed	0.74 (0.42, 1.07)	<0.00001
NK	3	264	94%	<0.00001	SMD, Random	0.24 (−0.77, 1.25)	0.65

*Inflammation factor*							
IL-1	4	302	98%	<0.00001	SMD, Random	−0.15 (−2.1, 1.8)	0.88
IL-8	3	252	95%	<0.00001	SMD, Random	−1.66 (−2.99, −0.33)	0.01

*Organ function*							
ALT	3	252	98%	<0.00001	SMD, Random	−4.85 (−8.13, −1.57)	0.004
AST	3	252	0%	0.97	SMD, Fixed	−6.13 (-6.73, −5.53)	<0.00001
BUN	3	252	87%	0.0004	SMD, Random	−1.63 (−1.92, −1.34)	<0.00001
Cr	5	375	98%	<0.00001	SMD, Random	−2.71 (−4.79, −0.64)	0.01
LDH	2	172	36%	0.21	SMD, Fixed	−2.00 (−2.45,−1.5)	<0.00001
CK	4	358	96%	<0.00001	SMD, Random	−1.57 (−2.82, −0.33)	0.01
CK-MB	7	513	84%	<0.00001	SMD, Random	−1.07 (−1.55, −0.59)	<0.0001
BNP	4	261	42%	0.16	SMD, Fixed	−0.45 (−0.69, −0.20)	0.0004
TnI	3	198	29%	0.24	SMD, Random	−0.67 (−1.02, −0.31)	0.0003

*Others*							
WBC	3	180	0%	0.76	SMD, Fixed	−0.11 (−0.41, 0.18)	0.44
Hb	3	163	0%	0.78	SMD, Fixed	14.59 (9.7, 19.48)	<0.00001

*Note.* No., number; EG, experimental group; CRP, C-reaction protein; IL-6, interleukin-6; NK, natural killer; ALT, alanine transaminase; AST, aspartate transaminase; BUN, blood urea nitrogen; Cr, creatinine; LDH, lactate dehydrogenase; CK, creatine kinase; CK-MB, creatine kinase isoenzyme-MB; APTT, activated partial thromboplastin time; PT, prothrombin time; TT, thrombin time; FIB, fibrinogen; PLT, platelet; D-D, D-dimer; IL-1, interleukin-1; TNF-*α*, tumor necrosis factor-*α*; IL-8, interleukin-8; WBC, white blood cell; Hb, hemoglobin; BNP, B-brain natriuretic peptide; TnI, troponin I.

## Data Availability

All data generated or analyzed during this study are included in this published article.
